RETRACTED

# Porosity Defect Remodeling and Tensile Analysis of Cast Steel

**DOI:** 10.3390/ma9020119

**Published:** 2016-02-22

**Authors:** Linfeng Sun, Ridong Liao, Wei Lu, Sibo Fu

**Affiliations:** 1 School of Mechanical Engineering, Beijing Institute of Technology, Beijing 100081, China; sunlinfeng1986@163.com; 2 Department of Mechanical Engineering, University of Michigan, Ann Arbor, MI 48109, USA; weilu@umich.edu; 3 Art and Science School, Eastern Michigan University, Ypsilanti, MI 48197, USA; yli18@emich.edu

**Keywords:** cast steel, porosity, mapping, radiographic, simulation

## Abstract

Tensile properties on ASTM A216 WCB cast steel with centerline porosity defect were studied with radiographic mapping and finite element remodeling technique. Non-linear elastic and plastic behaviors dependent on porosity were mathematically described by relevant equation sets. According to the ASTM E8 tensile test standard, matrix and defect specimens were machined into two categories by two types of height. After applying radiographic inspection, defect morphologies were mapped to the mid-sections of the finite element models and the porosity fraction fields had been generated with interpolation method. ABAQUS input parameters were confirmed by trial simulations to the matrix specimen and comparison with experimental outcomes. Fine agreements of the result curves between simulations and experiments could be observed, and predicted positions of the tensile fracture were found to be in accordance with the tests. Chord modulus was used to obtain the equivalent elastic stiffness because of the non-linear features. The results showed that elongation was the most influenced term to the defect cast steel, compared with elastic stiffness and yield stress. Additional visual explanations on the tensile fracture caused by void propagation were also given by the result contours at different mechanical stages, including distributions of Mises stress and plastic strain.

## 1. Introduction

Defects of cast steel, like shrinkage cavity and porosity, are always the common interferences to the material property and sometimes difficult to eliminate completely. Nowadays, effects of voids on the mechanical performance of castings have been widely investigated under different length scales. It is found that microscopic voids may not result in an evident loss of material stiffness, or large stress concentrations in a short life period. However, they can decrease the ductility of cast steel [1,2] at measurable levels. Although variously optimal casting technologies have been applied, macro-porosity can still be found in the structure. These non-uniformly distributed defects do not only cause the gross section loss and weaken the effective stiffness [3,4,5], but also make the material heterogeneous. 

RETRACTED

According to the porosity levels, porous materials can be classified into three categories: more than 70%, 10% to 70% and less than 10%. Mechanical models of the high-percentage category, which are usually foam and cellular materials [6], cannot be used in cast steels, because the basic assumption is totally different. When dealing with the low-percentage category, it is always assumed that voids are isolated from each other [7], or uniformly distributed [8]. Stiffness is considered to be linear with porosity, and “Porous metal plasticity” model, which has already existed in ABAQUS (ABAQUS Inc., Provindence, RI, USA), can appropriately describe the plastic behavior and failure. As for the mid-percentage category, current mechanical models now still cannot be unified due to the strongly non-linear dependency on porosity [9]. The study performed in this paper was to explore the possibility of predicting mechanical behavior of cast steel containing void defects regardless of the porosity levels. As an important tool, radiographic inspection technique could make great contributions during the analysis procedure.

To make the porosity prediction accurate and reliable, non-destructive evaluation (NDE) has become the method of preference among the engineers to investigate the inner-defect distributions in the cast steels [10,11,12]. By using computer tomography and scanning electron microscope (SEM) technique, Ries [13] claimed an approach to predict the porosity influence on material properties of cast alloys. In this way, actual defect morphologies could be captured and remodeled with finite elements. Although this work made great advances on multi-scale method, it basically focused on the microscopic unit cell modeling. Confronting with the non-uniformly distribution and large amount of porous defects under different length scales, this method still had some limitations.

In this paper, finite element method was combined with radiographic inspection technique in order to enlarge the usable length scale. Elastic behavior dependence on porosity is presented in Section 2, as is the Gurson-Tvergaard-Needleman (GTN) model being used to describe the plastic performance. In Section 3, cast steel specimens containing centerline porosity were made by ASTM A216 [14] WCB steel, and detailed sizes were also presented. After applying radiographic inspection, defect morphology data were mapped to the finite element (FE) model and the computational model for the specimen containing defects had been remodeled. In Section 4, ABAQUS input parameters were confirmed by trial simulations to the matrix specimen and comparison with experimental outcomes. It was found that simulation result data had good agreements with the measured data, and the claimed approach could provide correct predictions of the fracture positions. Conclusions were summarized in Section 5.

RETRACTED

## 2. Mathematical Model Analysis

In this paper, the mechanical property in elastic stage is considered as the function with porosity fraction f,$f=V_{void}/V_{0}$, where $V_{void}$ is the total volume of the voids in the material, $V_{0}$ is the total volume of the material. The elastic behavior then could be observed by the variation of porosity fraction field. Both elastic modulus *E* and Possion ratio υ are dependent on porosity *f* and relevant equations are given as follows [4,15,16]:

(1) $$\left\{ \begin{array}{l} E(f)=E_{0}{\left(1-f/0.5\right)}^{2.5}\\ \nu (f)=\nu_{0}+\left(f/0.472\right)\left(0.14-\nu_{0}\right) \end{array}\right.$$

According to the ASTM standard values of WCB cast steel, *E*_0_ = 198,000 MPa, υ_0_ = 0.3. When using porous metal plasticity, relation between yield stress and plastic strain of the matrix material should be developed first. Specifically, the hardening curve which is shown in Figure 1 is determined from tensile test for the WCB matrix steel.

As a readily available constitutive model to investigate the effect of porosity on casting’s fracture behavior, the GTN plasticity model has been used in this study. The complete description of this model can be found in Gurson’s work [17,18]. The yield condition of the porous material can be concluded as follows, where *f* is the porosity fraction, *q* is the effective Mises stress, *p* is the hydrostatic stress, σ*_y_* is the yield stress of the matrix material as a function of plastic strain, $q_{1}$, $q_{2}$ and $q_{3}$ are material parameters.

(2) $$\phi ={\left(q/\sigma_{y}\right)}^{2}+2q_{1}f\cosh\left(-3q_{2}p/2\sigma_{y}\right)-\left(1+q_{3}f^{2}\right)=0$$

Note that Equation (2) could become Mises yield condition when f=0. p and q are two stress invariants, whose formulas are p=−(1/3)σ:I and $q=\sqrt{\left(3/2\right)S:S}$, respectively. σ is Cauchy stress tensor, S is deviatory stress tensor, S=pI+σ. The material parameters $q_{1}$, $q_{2}$ and $q_{3}$ are related to the interaction between voids [8], which are set to 1.5, 1.0 and 2.25. Flow rules for the plastic strain rate ${\dot{\varepsilon }}^{pl}$ is shown below:

(3) $${\dot{\varepsilon }}^{pl}=\dot{\lambda }\left(\partial \phi /\partial \sigma \right)=\dot{\lambda }\left[\left(3/2q\right)\left(\partial \phi /\partial q\right)S-\left(1/3\right)\left(\partial \phi /\partial p\right)I\right]$$

where $\dot{\lambda }$ is a non-negative scalar constant, it is used to measure the plastic flow rate. With the increase of plastic strain, void nucleation and propagation will be induced until material damage. This phenomenon can be described by using the growth rate equation of voids, $\dot{f}=\left(1-f\right){\dot{\varepsilon }}_{kk}^{pl}+A{\dot{\varepsilon }}_{m}^{pl}$.

RETRACTED

The first term on the right-hand side represents existing void propagation with current porosity fraction f and total plastic strain rate ${\dot{\varepsilon }}_{kk}^{pl}$, which is the trace of the strain rate tensor. The second term represents porosity fraction growth rate because of the void nucleation. $A=\left(1/s_{N}\sqrt{2\pi }\right)f_{N}\exp\left[-{\left(\varepsilon_{m}^{pl}-\varepsilon_{N}\right)}^{2}/\left(2s_{N}^{2}\right)\right]$, is a scaling coefficient [18], ${\dot{\varepsilon }}_{m}^{pl}$ is the equivalent plastic strain rate. In this paper, the mean value of plastic strain $\varepsilon_{N}=0.3$, standard deviation $s_{N}=0.1$, porosity fraction of nucleated voids $f_{N}=0.04$.

Considering the coalescence after void growth, Needleman [19] claimed a void coalescence and failure criteria theory, which replaced f with effective porosity fraction $f^{*}$. The specific equation set is as follows:

(4) $$f^{*}=\left\{ \begin{array}{cc} f, & f\leq f_{c}\\ f_{c}+\left({\bar{f}}_{F}-f_{c}\right)\left(f-f_{c}\right)/\left(f_{F}-f_{c}\right), & f_{c}<f\leq f_{F}\\ {\bar{f}}_{F}, & f>f_{F} \end{array}\right.$$

where $f_{c}$ is the critical fraction when the void interaction begins, $f_{F}$ is the failure fraction when the material fracture begins, ${\bar{f}}_{F}$ is related with material parameters $q_{1}$ and $q_{3}$, ${\bar{f}}_{F}=\left(q_{1}+\sqrt{q_{1}^{2}-q_{3}}\right)/q_{3}$. In this paper, $f_{c}=0.05$ and $f_{F}=0.15$.

## 3. Experiments and Simulation Model

### 3.1. Selection of Specimen Structure and Material

To investigate the mechanical property influences brought by irregular void defects, cast steel specimens containing centerline porosity were made by ASTM A216 WCB steel. After being normalized and tempered, cast blanks were machined into specimens according to the ASTM E8 [20] tensile test standard, detailed sizes were shown in Figure 2a. 

To keep generality, the specimens were divided into two groups: Height = 457 mm (named as Group A) and Height = 381 mm (named as Group B), each group had 5 specimens. Besides, two small specimens, which were presented in Figure 2b, had been 1/9 cut from the void-free sections from the cast blanks. These two specimens were used to gain the tensile values of matrix material, like elastic modulus $E_{0}$, yield stress $\sigma_{y0}$, ultimate strength and elongation.

RETRACTED

### 3.2. Radiograph Analysis and Finite Element Remodeling

Through radiographs of specimens, void characteristics and distributions could be specified by the gray density levels, which were shown in Figure 3a. These photos were taken 10 pixels per mm. The yellow rectangle includes the stepped gray bars and the thickness of the specimen would decrease when the bar became darker. In this paper, the gray levels which were higher than 0.75 (representing thickness equal to 19.1 mm) would not be considered. Meanwhile, gray levels which were under 0.31 (representing thickness equal to 7.9 mm) could not be captured due to the limits of test instrument.

After removing the disturbances (shadow *etc.*), only the pixels specified as void defects could be used for the thickness analysis; otherwise the pixels were considered as matrix material. Thickness value in each pixel was divided by the total thickness (19.1 mm), and then porosity fraction in each pixel could be obtained. The minimum porosity fraction for this study was approximately 1.5%. The complete procedure was summarized in Figure 3a–d, accordingly.

The fracture photograph for the specimen A3 was shown in Figure 4a with the actual fracture location being identified by the red box. When dealing with the original radiograph of A3 (Figure 4b), porosities on different cross sections being normal to the tensile direction were measured along the specimen length. When they were above the mid-length, the distance values were positive, and the negative ones were below the mid-length. Data in Figure 4c indicated the various cross section porosities at different distances from the mid-length. It seemed that the averaged value was 0.19% and the maximum value was around 0.80%, which had fell into the fracture section. This phenomenon indicated that the fracture location could easily correspond with the region of high cross section porosity. 

The porosities on the fracture surfaces were measured to make an appropriate assumption for the porosity thickness used in the following simulations. Figure 4d presented the fracture surface of the specimen A3 and it can be observed that all the void defects were basically centerline type. After checking all the fracture surfaces, it had been observed that the maximum vertical value of porous region that caused fracture was approximately 2.2 mm.

Then porosity fraction data from the distribution contour (*i.e.*, Figure 3a) was mapped to the relevant mesh nodes assuming that it lay symmetrically on the centered thickness plate in the 2.2 mm region, corresponding to the two center-most elements on each side of the specimen. The transfer procedure was managed by computer code. The refined mesh model and porosity mapped model could be found in Figure 5a,b. The average porosity on the nodal spacing was calculated by interpolation method in order to conserve the porosity data from the radiograph. Because each node was shared with multiple elements, the porosity field appeared to diffuse beyond the two center-most elements. After mapping and remodeling of the porosity fraction field, further simulations could be engaged in ABAQUS/Explicit with relevant boundary conditions.

RETRACTED

## 4. Experimental and Simulation Results and Comparison

### 4.1. Experimental Results of Tensile Tests

Stress-strain curves extracted from the tests on matrix WCB and porous WCB specimens were presented in Figure 6a. Figure 6b indicated the detailed results when strains were ended up to 0.04, and it mainly focused on the elastic stages and yield stress points. Detailed result data of all 11 specimens were listed in Table 1. It could be observed that the data from matrix WCB specimen basically coincided with the ASTM A216 WCB standard values.

From Figure 6b, all 10 defect specimens had shown various non-linear trends and relevant stiffness had also decreased accordingly. This phenomenon was believed to be caused by non-uniformly distributed stress and local yielding around inner voids. In order to obtain the elastic modulus, chord modulus [21] was introduced to involve in the calculation with stress and strain values at 10% and 90% of the yield stress.

If the cast condition remained the same, the higher specimen would produce a higher possibility to misrun. Then the mechanical property would weaken with no doubt. After the tests, it could be seen that four of the five highest-elastic-modulus specimens were from the ones that had larger heights. The same phenomenon happened in the yield stress cases. Noted that five specimens who had the highest elastic modulus were named as A1 to A5, the rest were B1 to B5, accordingly.

### 4.2. Simulation Results of Tensile Tests

As was mentioned above, some micro voids, which were under the capture limit of test instrument, still existed in the specimens. So the initial porosity fraction $f_{0}$ might be under-evaluated if they were only defined from radiographs. After series of tensile simulations and comparisons with experimental data, $f_{0}$ was finally selected as 0.002. Relevant comparison curves were presented in Figure 7 and detailed input parameters used in ABAQUS were listed in Table 2.

It could be indicated from Figure 8 that the simulation results had good correspondence with the experimental curves. The inner defects had minus effects on elastic stiffness. However, these voids could have an obvious impact on the tensile failure, and the prediction for the fracture positions from FE simulations also basically fitted with the tensile tests. As for the simulation errors, they was due to the incomplete mapping for all the void defects in the specimens, or the data lost during the mapping procedure.

RETRACTED

Detailed simulation result data of all 11 specimens were listed in Table 3. Compared with Table 1, the computation errors stayed in the acceptable range. Note that the elongation simulation results of samples B1 and B4 did not have good agreements with the experimental values. This discrepancy might be due to the equipment’s tensile velocity abnormal changes during the yielding period. This variation could disturb the locations of inflection point of stress at the tensile curves, or make the software provide incorrect judgments of the yielding period’s end point. Figure 9 showed the fracture positions in both experiments and simulation predictions, and it was observed that the finite element models could provide mostly accurate predictions to the tensile fracture positions.

To investigate the failure procedure with porosity variation more deeply, specimen A3 was selected as the sample. Mises stress and plastic strain values were examined at Point A, B and C, which were shown in Figure 10a and represented the strain values as 0.014, 0.045 and 0.104, respectively. Porosity propagation at the three mentioned stages could be observed in Figure 10b. Because of $f_{F}=0.15$, the maximum scale for the porosity fraction was set to 0.15. It could be seen that two condensed void-gathering sections had emerged, and they would provide the possibility to make a fracture. 

Figure 10c presented the Mises stress contours at the three points. Note that even at the elastic stage, stress in some areas could still go beyond the yield limit. It was observed that the porous area carried no stress at all. The upper void-gathering section had more serious plastic deformation problems, which could be seen in Figure 10d, and that was the reason why tensile fracture happened there first. All these results were exhibited at mid-stiffness slices, and they were hoped to give more detailed information on exploring mechanical behaviors of defect casting materials.

As was presented in Figure 11, solid and dashed curves demonstrated the simulated development of averaged porosity and Mises stress with the strain values of specimen A3 during the tension period, respectively. The initial averaged porosity fraction was about 0.75% and increased slowly until reaching the ultimate tensile stress, then rapidly increased due to the failure event. This result could provide additional insight into the interaction between porosity and mechanics.

RETRACTED

## 5. Conclusions

The current work demonstrates that the tensile fracture of cast steel material with porous defects can be predicted from radiographs by using porosity mapping and reconstruction in the finite element analysis (FEA) software. Porous metal plastic constitutive model, which is commonly implemented in ABAQUS, has been applied to describe the mechanical behavior. The most noticeable influence brought by porosity is reduction in ductility, with the elongation ranging from 12.80% to 19.60% *versus* 22.00% for the matrix steel. Although two of 10 simulated elongations have singularities, the rest show good agreement with the measured results in general. The maximum error is 1.50% and the minimum one is 0.10%, and this error range seems acceptable to the computation.

The evolution of porosity inside the specimen during the tensile procedure can also be revealed in order to investigate the failure procedure with porosity variation more deeply. Coupled with the stress and strain distribution contours, the location of tensile fracture can be predicted by simulation and the result is in accordance with the test.

It should be noticed that some disagreements still remain between simulation and measured results. Neglecting the experimental instrument issues, the possible reasons to the errors maybe due to the limitations of the porous metal plasticity model, or the assumptions and deficiencies in prescribing the porosity thickness scales of the specimens. The method described in this paper can be improved by more realistic porosity reconstruction techniques, like tomography. In other words, the more accurate porosity distribution inputs used in the simulation, the more precise prediction results we can get. This is also the future work which the authors are planning to do.

## Figures and Tables

**Figure 1:** Hardening curve of the matrix material.

**Figure 2:** Experimental specimen and cast blank radiograph: (**a**) Dimensions of the specimen; (**b**) Selecting location of the matrix specimen.

**Figure 3:** Porosity fraction result: (**a**) Original radiograph; (**b**) Image of defect after shadow filtration; (**c**) Thickness distribution in the specimen; (**d**) Porosity fraction field distribution.

**Figure 4:** Images of tensile fracture location and initial porosity analysis of specimen A3: (**a**) Fracture location of A3; (**b**) Radiograph of porosity distribution along different distances from mid-length; (**c**) Cross section porosity distribution curve; (**d**) Fracture surface of A3.

**Figure 5:** Finite element (FE) mapping model: (**a**) Meshing details; (**b**) Computational FE model after mapping and remodeling.

RETRACTED

**Figure 6:** Tensile test curves of the 11 specimens: (**a**) Complete tensile test curves for all specimens; (**b**) Stress-strain curves after scaling up for all specimens.

**Figure 7:** Tensile result comparison of the matrix specimen between test and simulation. (**a**) Complete tensile result curves; (**b**) Curves after scaling up.

**Figure 8:** Tensile result comparisons of the defect-containing specimens between test and simulation: (**a**) Specimen B1; (**b**) Specimen B2.

**Figure 9:** Comparisons of the fractures between test and simulation predicting: (**a**) Specimen A2; (**b**) Specimen A3.

**Figure 10:** Tensile performance on Specimen A3: (**a**) Locations of 3 examiningpoints (A, B and C), which represent different stages of strain; (**b**) Porosity propagation contours at three examining points (A, B and C); (**c**) Stress propagation contours; (**d**) Plastic strain propagation contours at three examining points (A, B and C).

**Figure 11:** Simulated development of averaged porosity and Mises stress with strain of Specimen A3.

**Table 1:** Tensile test results for all specimens.

Specimen	Elastic Modulus (MPa)	Yield Stress (MPa)	Ultimate Strength (MPa)	Elongation (%)
A1	179,931.92	351.71	573.65	16.11
A2	179,649.23	388.53	575.66	16.30
A3	178,766.67	362.13	525.68	13.80
A4	174,167.70	375.02	554.43	12.80
A5	173,126.56	383.71	572.63	16.00
B1	172,175.05	355.30	532.09	15.00
B2	169,051.61	349.23	543.88	17.00
B3	162,625.47	368.06	562.08	13.80
B4	157,178.42	329.24	542.02	19.60
B5	137,258.77	373.36	575.80	17.10
Matrix	190,302.00	356.89	556.08	22.00

**Table 2:** Setup for the simulation parameters.

$q_{1}$	$q_{2}$	$q_{3}$	$f_{0}$	$f_{c}$	$f_{F}$	$\varepsilon_{N}$	$s_{N}$	$f_{N}$
1.5	1	2.25	0.002	0.05	0.15	0.3	0.1	0.04

**Table 3:** Tensile simulation results for all specimens.

Specimen	Yield Stress (MPa)	Ultimate Strength (MPa)	Elongation (%)
A1	359.22	568.97	16.23
A2	380.37	565.19	16.15
A3	339.23	524.02	12.30
A4	380.30	535.33	11.89
A5	375.27	560.91	16.10
B1	352.33	538.50	10.70
B2	337.17	533.67	16.20
B3	356.37	533.67	13.90
B4	346.82	536.43	11.80
B5	355.82	555.74	17.00
Matrix	350.27	555.74	21.50
